# Macrophage Colony-Stimulating Factor Augments Tie2-Expressing Monocyte Differentiation, Angiogenic Function, and Recruitment in a Mouse Model of Breast Cancer

**DOI:** 10.1371/journal.pone.0098623

**Published:** 2014-06-03

**Authors:** Mary A. Forget, Jeffrey L. Voorhees, Sara L. Cole, Duaa Dakhlallah, Ivory L. Patterson, Amy C. Gross, Leni Moldovan, Xiaokui Mo, Randall Evans, Clay B. Marsh, Tim D. Eubank

**Affiliations:** 1 Department of Internal Medicine, Division of Pulmonary, Allergy, Critical Care, and Sleep Medicine, The Ohio State University, Columbus, Ohio, United States of America; 2 Molecular Cellular and Developmental Biology Program, The Ohio State University, Columbus, Ohio, United States of America; 3 Campus Microscopy and Imaging Facility, The Ohio State University, Columbus, Ohio, United States of America; 4 The Center for Biostatistics, The Ohio State University, Columbus, Ohio, United States of America; 5 The Ohio State University Comprehensive Cancer Center, The Ohio State University, Columbus, Ohio, United States of America; University of Barcelona, Spain

## Abstract

Reports demonstrate the role of M-CSF (CSF1) in tumor progression in mouse models as well as the prognostic value of macrophage numbers in breast cancer patients. Recently, a subset of CD14+ monocytes expressing the Tie2 receptor, once thought to be predominantly expressed on endothelial cells, has been characterized. We hypothesized that increased levels of CSF1 in breast tumors can regulate differentiation of Tie2- monocytes to a Tie2+ phenotype. We treated CD14+ human monocytes with CSF1 and found a significant increase in CD14+/Tie2+ positivity. To understand if CSF1-induced Tie2 expression on these cells improved their migratory ability, we pre-treated CD14+ monocytes with CSF1 and used Boyden chemotaxis chambers to observe enhanced response to angiopoietin-2 (ANG2), the chemotactic ligand for the Tie2 receptor. We found that CSF1 pre-treatment significantly augmented chemotaxis and that Tie2 receptor upregulation was responsible as siRNA targeting Tie2 receptor abrogated this effect. To understand any augmented angiogenic effect produced by treating these cells with CSF1, we cultured human umbilical vein endothelial cells (HUVECs) with conditioned supernatants from CSF1-pre-treated CD14+ monocytes for a tube formation assay. While supernatants from CSF1-pre-treated TEMs increased HUVEC branching, a neutralizing antibody against the CSF1R abrogated this activity, as did siRNA against the Tie2 receptor. To test our hypothesis *in vivo*, we treated PyMT tumor-bearing mice with CSF1 and observed an expansion in the TEM population relative to total F4/80+ cells, which resulted in increased angiogenesis. Investigation into the mechanism of Tie2 receptor upregulation on CD14+ monocytes by CSF1 revealed a synergistic contribution from the PI3 kinase and HIF pathways as the PI3 kinase inhibitor LY294002, as well as HIF-1α-deficient macrophages differentiated from the bone marrow of HIF-1α*^fl/fl^*/LysMcre mice, diminished CSF1-stimulated Tie2 receptor expression.

## Introduction

Macrophage colony-stimulating factor (CSF1) drives the survival and differentiation of monocytes, recruited from the bone marrow, to macrophages [1]. Upon binding to the CSF1R (CSF1R/c-fms), CSF1 causes receptor dimerization and phosphorylation of tyrosine kinase sites on the intracellular domain of the receptor. Phosphorylation of the intracellular domain of CSF1R results in activation of intracellular signal transduction pathways involving PI3 Kinase-Akt, Ras/MAPK, Stat-1 and -3, Jak1, Phospholipase A2 and 1C, and these activation regulates numerous cellular events that facilitate an innate immune response [2]–[6].

Tumor-associated macrophages (TAMs) arise from peripheral blood monocytes that diapedes through the endothelial barrier in response to chemoattractant signals released during an inflammatory response or by neoplastic and tumor stromal cells [7]–[9] and this extravasation into tumor tissue is accompanied by, and coordinated with, the differentiation of monocytes into macrophages [10], [11]. Tumor macrophages can have either a positive or negative effect on tumor cell proliferation. Macrophages exert anti-tumor effects through cytotoxic killing of tumor cells and presentation of tumor antigens [12]. As transformed cells develop into tumor tissue, “tumor-helping” tumor-associated macrophages (TAMs) facilitate tumor growth and progression through the production of proteases and angiogenic factors [13], [14]. In patient studies, increased numbers of macrophages correlate with poor prognosis in human breast carcinomas [15]. As the tumor progresses, macrophage differentiation is skewed towards an anti-inflammatory M2 phenotype. These alternatively-activated macrophages function in the tissue repair process through production and expression of IL-10, arginase-1, TGF-β, and mannose receptor [16], [17]. In addition, M2 macrophages produce factors that facilitate angiogenesis [18], [19]. For example, treatment of macrophages with CSF1 up-regulates the potent pro-angiogenic molecule vascular endothelial growth factor (VEGF) which increases endothelial cell proliferation and migration to drive new blood vessel growth [13]. Production of these factors has been demonstrated in solid tumors, such as breast cancer, where CSF1 increases angiogenic branching and blood vessel density. In mouse models, mice deficient in CSF1 have reduced vessel density and fewer tumor metastases than mice producing normal levels of CSF1 [20], [21]. Moreover, the re-introduction of CSF1 locally into the tumor restores the tumor macrophage population, tumor vessel density, and metastasis [20].

Recently, a subpopulation of M2 macrophages which express endothelial cell tyrosine kinase receptor, Tie2, has been identified [22], [23]. These Tie2-expressing monocytes/macrophages (TEMs) are major contributors to tumor angiogenesis, progression and metastasis [24]–[26]. For example, co-injection of isolated TEMs with glioma cells in mice increases tumor angiogenic area [23]. Myeloid-specific knockdown of Tie2 via miRNA decreases tumor volume and tumor cell metastasis to the lung [26], [27]. Further, antibody therapy blocking the Tie2 ligand, Angiopoietin-2 (ANG2), results in decreased tumor angiogenesis and progression [26]. *In vitro* studies support the pro-angiogenic role of TEMs and a gene expression profile that resembles, but does not completely overlap, M2 macrophages. In tube formation assays, the conditioned media from TEMs produced more branch points than Tie2 receptor negative monocytes [28]. IL-10 produced by monocytes following ANG2 treatment suppresses tumor immunity by decreasing T cell proliferation and cytotoxicity [29]. TEMs also produce high amounts of remodeling factors, such as MMP-9 and thymidine phosphorylase, facilitating macrophage migration to hypoxic and necrotic areas [28].

In summary, we observed that CSF1 treatment augments Tie2 receptor expression on CD14+ human monocytes in culture. Further, pre-treatment of CD14+ monocytes with CSF1 induced cell migration in response to ANG2 as well as augmented the angiogenic potential on HUVEC when cultured in cell-free supernatants from these TEMs while a neutralizing antibody for CSF1R, or siRNA against Tie2 receptor, abrogated this effect. To illustrate the relevance of this phenomenon *in vivo*, we treated PyMT breast tumor-bearing mice with CSF1 and analyzed bone marrow, peripheral blood, and tumors for changes in TEM population compared to total macrophages. While CSF1 did not induce an increase in the TEM precursors in bone marrow, we did observe an increase in each peripheral blood and tumor TEMs compared to total monocyte/macrophage populations. Finally, using bone marrow-derived macrophages from wild type LysMcre or HIF-1α*^fl/fl^*LysMcre mice, we report that CSF1-induced expression of Tie2 receptor is regulated by a synergistic contribution of the PI3 kinase and HIF pathway in an oxygen-independent manner. The importance of this study is highlighted by our data suggesting that high serum levels of CSF1 in breast cancer patients may be responsible for increasing the number of circulating monocytes recruited to tumors and their support of tumor progression.

## Materials and Methods

### Ethics Statement

This study was carried out in strict accordance with the recommendations in the Guide for the Care and Use of Laboratory Animals of the National Institutes of Health. The animal protocols were approved by the Institutional Laboratory Animal Care and Use Committee (ILACUC) of the Ohio State University (protocols: 2011A00000077 and 2009A0124-R1). The Ohio State University Institutional Review Board approved both the written consent procedure and this study for the collection and use of human monocytes isolated from peripheral blood of healthy volunteers. The volunteer blood donors gave written consent to be included in this study.

### Monocyte Isolation

Peripheral blood mononuclear cells were isolated by a Ficoll gradient and CD14+ monocytes were collected by positive bead separation as per manufacturerXC's protocol (Miltenyi Biotech). Isolated CD14+ monocytes (2×10^6^) were incubated in endotoxin-free RPMI media (BioWhittaker) with 1% FBS (certified as containing <0.06 EU/ml endotoxin levels from HyClone, Logan, UT), penicillin (100 U/ml), streptomycin (100 U/ml), amphotericin B (0.25 µg/ml) (Gibco) and 10 µg/ml polymyxin B (Calbiochem).

### Flow Cytometry

Freshly-isolated CD14+ human monocytes were incubated for specified times. The cells were incubated with media containing rhANG1 (100 ng/ml), rhANG2 (100 ng/ml), rhCSF1 (0.1, 1, 10, or 100 ng/ml), or pre-treated with media containing a neutralizing antibody targeting the CSF1R (R&D Systems clone 61701). The cells were fixed then blocked with anti-FcγR antibody (R&D System) for 15 minutes at 4°C to prevent non-specific binding. Cells were incubated with 10 µl PE-conjugated anti-human Tie2 (clone 83715, R&D Systems) per 1×10^6^ cells at 4°C for 30 minutes per manufactures instructions or 10 µl of the isotype control PE-conjugated anti-human IgG (R&D Systems). Tie2-expressing monocytes were subsequently analyzed using the Aria III flow cytometer at The Ohio State University Flow Cytometry Core Facility.

### Migration Assay

CD14+ human monocytes were isolated as described above and cultured in RPMI media containing 1% FBS without or with 10 ng/ml rhCSF1 in the bottom well of Boyden chemotaxis chambers for 18 hours. The cells were washed 3× with PBS and the media replaced with FBS-containing RPMI without or with a dose escalation of rhANG2 (0.1, 1, 10, 100, 300 ng/ml) in the top chamber. After 24 hours, the filters were inspected for monocytes which migrated to the top chamber (chemotaxis) and blindly counted by microscopy. In another experiment, CD14+ monocytes were treated as above except transfected with 25, 50, or 100 nM scrambled siRNA-GFP conjugate or siRNA-GFP targeting the human Tie2 receptor (Santa Cruz) (*Figure S2*). The cells were washed and sorted using flow-assisted cell sorting for GFP expression to confirm successful transfection followed by Boyden chamber chemotaxis assay as described above.

### HUVEC Branching Assay

CD14+ human monocytes were cultured in RPMI media containing 1% FBS alone or in combination with rhVEGF (10 ng/ml), rhCSF1 (10 ng/ml), or rhANG2 (10 ng/ml) for 18 hours followed by 3 PBS washes and subsequent incubation in ANG2 (10 ng/ml)-containing media for 24 hours. The cell-free supernatants were collected by centrifugation. 5×10^3^ HUVEC (ATCC) per well in a 24 well plate were cultured on top of 120 µls growth factor-reduced Matrigel (BD Discovery Labware) in the cell-free conditioned supernatant. The HUVECs were cultured for 6 hours in these conditioned supernatants and branch points counted in a blinded manner. In another experiment, CD14+ monocytes were pre-treated with a neutralizing antibody against CSF1R (40 µg/ml) for 30 minutes before 18 hours incubation with rhCSF1 (10 ng/ml), 3 PBS washes, and ANG2 treatment (10 ng/ml) for 24 hours. In another experiment, CD14+ monocytes were treated as above except transfected with a scrambled siRNA-GFP conjugate or siRNA-GFP targeting the human Tie2 receptor. The cells were washed and sorted using flow-assisted cell sorting for GFP expression to confirm successful transfection followed plating and collection of conditioned supernatants as described above.

### Real-time PCR

CD14+ monocytes were subjected to Trizol reagent (Invitrogen). RNA was extracted in chloroform and purified using the RNeasy Mini kit (Qiagen). cDNA was generated from 1 µg of RNA using the Superscript First Strand Synthesis System (Invitrogen) and reactions performed using SYBR Green PCR Master Mix (Applied Biosciences) according to the manufacturer's instructions. See *Table S1* for list of primers used in this st udy. Data were analyzed according to the comparative threshold method and normalized against the GAPDH internal control transcript.

### CSF1R Neutralization *In Vivo*

Inhibition of the CSF1R on CD14+ human monocytes was accomplished with a neutralizing antibody targeting the CSF1R (R&D Systems clone 61701). For neutralization of the CSF1R in mouse PyMT breast tumors, 50 mg/kg body weight of ASF98 rat anti-mouse monoclonal *c-fms* antibody was used. Dr. Shin-Ichi Nishikawa kindly provided the ASF98 hybridoma (Riken Center for Developmental Biology, Kobe, Japan). Antibodies were produced and isolated as previously described [30], [31]. Briefly, hybridoma cells were grown in serum-free media (Gibco) until the media exhausted. Cell-free supernatant was collected by centrifugation and loaded onto a protein A/G agarose bead column. Antibody was then eluted using elution buffer (Thermo Scientific). Elution fractions were neutralized with 1.5 M Tris base (pH 8.0) and pooled fractions were concentrated by centrifugation through concentration columns (Millipore). Antibody concentration was determined using the Bradford colorimetric assay and samples compared to BSA protein standards.

### PyMT Tumor Model

PyMT tumor cells from C57Bl/6 mice were cultured in Dulbecco's Modified Eagles Medium (DMEM) supplemented with 1% PSA, 10% FBS, 10 µg/ml human insulin, and 5 µg/ml rmEGF. Tumor cells (1×10^6^ cells in 100 µl) were injected orthotopically into the number four mammary fat pad of naïve 6–8 week old female C57Bl/6 wild type mice or C57Bl/6 LysMcre or HIF-1α*^fl/fl^*/LysMcre mice. Beginning with palpation (about 2 weeks post-injection), tumor growth was measured 3 times per week using calipers and tumor volume calculated using the equation: Tumor volume  = 0.5× [(large diameter) × (small diameter)^2^]. In one study, the tumors were treated when palpable with 50 µls of PBS, CSF1R NAb (50 mg/kg), or IgG Ab (50 mg/kg). Four hours later, the tumors were injected with 50 µls PBS or rmCSF1 (100 ng/ml). This treatment paradigm was delivered every other day for two weeks.

### Immunocytochemistry and confocal fluorescence microscopy

For confocal microscopy, 10 µm thick paraformaldehyde-fixed tumor tissue sections were incubated with antibody (1 µg/ml) to detect CD31 (rat anti-mouse, BD Pharmingen 553370), F4/80 (rat anti-mouse direct RPE label, Bio-Rad Laboratories, MCA497PE) and Tie2 (mouse anti-human, BD Pharmingen 557039). Fluorescence detection of Tie2 and CD31 was accomplished using Alexa Fluor 488 goat anti-mouse and Alexa Fluor 633 goat anti-rat antibodies respectively (Invitrogen, A11006 and A21094). DAPI was included to detect nuclei. Images were captured using an Olympus FV1000-Spectral Confocal system equipped with a PLAPONSC 60× oil-immersion objective lens (N.A. 1.4). Imaging for each fluorescence signal was performed either with or without a 3× optical zoom using the exact same detector settings in order to maximize signal-to-noise ratio. All presented images were processed identically using Adobe Photoshop CS5 software. For the “multiply overlay F4/80+/Tie2+” panels, the F4/80 only image was pasted beneath the Tie2 only image in a separate layer. The Tie2 only image was selected and the “multiply” option was applied. This feature enables the top image (Tie2 only) to act as a screen to allow the passage of the bottom layer (F4/80 only) to show through only where the top layer has positive pixels. Thus, the composite image illustrates where both Tie2 and F4/80 are positive in the same section.

### Tumor Cell Isolation

Age-matched PyMT tumor-bearing female C57Bl/6 mice were sacrificed by CO_2_ asphyxiation followed by cervical dislocation. Peripheral blood was removed by cardiac puncture. Bone marrow was isolated from the femurs and tumors harvested. Tumors were cut into small sections using a razor blade and enzymatically homogenized using 1 ml of PBS containing collagenase (0.55 mg/ml) and DNase (0.1 mg/ml). The tumors were incubated at 37°C and vortexed every 5 minutes for 30 minutes. Single cell suspensions were generated using 100 µm mesh cell strainers (Fisher Scientific) and washed twice with 10 ml PBS by centrifugation at 1500 rpm for 10 minutes. The mononuclear cell layer from peripheral blood and tumor homogenate was separated using a Ficoll gradient. The mononuclear cell layer was removed and washed twice with PBS. Any residual red blood cells were lysed using Red Cell Lysis Buffer (155 mM NH_4_Cl, 10 mM NaHCO_3_, 0.1 mM EDTA; pH = 7.4) for 5 minutes at room temperature. Bone marrow cells were centrifuged, resuspended in PBS and red blood cells lysed. Remaining cells were washed twice with PBS and resuspended in MACS buffer (Miltenyi Biotech). For flow cytometric analysis and cell sorting, cells isolated from tumors, peripheral blood and bone marrow were blocked with whole IgG for 15 minutes at 4°C. Samples were immunostained with antibodies specific for Tie2 receptor (PE-conjugate clone TEK4, eBiosciences), CD11b (Percy 5.5 and PE-conjugate clone M1/70), CD31 (PE-Cy7 and APC-conjugate clone 390), Gr-1 (Percy 5.5 and PE-conjugate clone RB6-8C5) (R&D Systems) and F4/80 (PE-Cy7 or APC-conjugate clone Cl:A3-1, Serotec). Isotype control samples were immunostained with rat anti-mouse IgG2_a_κ and IgG2_b_κ with corresponding fluorescent conjugates (R&D Systems). TEMs in this study are described as: CD45+/Tie2+ (bone marrow), CD11b+/CD31-/Gr-1^low^/Tie2+ (peripheral blood and tumor for comparing the different compartments), and F4/80+/Tie2+ (for comparative studies in tumor tissue by flow cytometry and immunohistochemistry). All flow cytometry was measured using the Aria III flow cytometer at The Ohio State University Flow Cytometry Core Facility.

### Tumor Angiogenesis

Tumors from PyMT tumor-bearing 6–8 week old female C57Bl/6 mice were collected at time of sacrifice as described above. Tumor sections were immunostained with CD31 antibody and imaged by fluorescent microscopy using a ×20 objective lens. Five random images per tumor per group were captured in a blinded manner, analyzed for CD31-positivity (red pixels), and quantified for red pixels per high powered field (HPF) of tissue using Adobe Photoshop CS2 (Adobe Systems) histogram analysis.

### Inhibitor studies

Macrophages were differentiated from the bone marrow of 6–8 week old female C57Bl/6 wild type mice LysMcre or C57Bl/6 HIF-1α*^fl/fl^*/LysMcre mice over five days using 20 ng/ml rmCSF1 in endotoxin-free RPMI, 1% FBS, and 10 µg/ml polymyxin B. The cells were pre-treated with the appropriate vehicle or the PI3 kinase inhibitor, LY294002 (50 µM), the MEK inhibitor, U0126 (10 µM), or the NF-κB inhibitor, PDTC (100 µM) for 30 minutes followed by stimulation with 100 ng/ml rmCSF1 or not for 24 hours. The cells were collected, fixed, and immunostained using F4/80 and Tie2 receptor antibodies as described above and subjected to flow cytometry for percent F4/80+/Tie2+ cells.

### Statistical Analyses

For assays determining effects of Tie2 expression by CSF1 on migration and HUVEC sprouting, the data was analyzed by linear mixed effect model which considers observational dependencies across treatments groups. For the assays determining percent TEMs or total F4/80+ cells in bone marrow, blood, or tumors, tumor volume determinations, small molecule inhibitor studies, and tumor angiogenesis, the data was analyzed by ANOVA. Holm's method was used to adjust multiplicity for primary comparisons when necessary. SAS 9.3 software was used for analysis (SAS, Inc. Cary, NC).

## Results

### CSF1 regulates a transition from CD14+ monocytes to CD14+/Tie2+ TEMs

CSF1 drives the differentiation of peripheral blood monocytes to macrophages resulting in a pro-angiogenic and immune regulatory phenotype [13], [32]. In breast tumors, CSF1 expression increases the number of macrophages which enhances tumor vessel density and metastasis [33]–[35]. Further, loss of CSF1 (*op/op* mice) hinders the development of tumor blood vessels and tumor progression [20]. Tie2-expressing monocytes/macrophages (TEMs) are a subset of myeloid cells that function similar to M2, tumor-associated macrophages (TAMs) as their activity increases tumor blood vessel area and metastasis in mouse models of breast cancer[24], [26], [27]. As stated above, CSF1 plays a role in normal mammary gland physiology and ductal development [21]. But, in breast cancer patients, CSF1 levels are augmented and predict poor outcome [15]. In 2003, we reported that CSF1 drove a pro-angiogenic phenotype in CD14+ monocytes via the production of VEGF [13]. However, in that study we did not consider that CSF1 may differentiation alternate subpopulations of monocytes. Thus, our current study examines a direct link between CSF1 and the expression of the Tie2 receptor on CD14+ human monocytes to become TEMs. To elucidate this effect, human monocytes were isolated from whole blood using CD14+ microbeads and incubated in non-adherent culture tubes in RPMI media containing fetal bovine serum and cultured for 24 hours with or without 100 ng/ml recombinant human CSF1. Even though lower doses can drive the differentiation, survival and function of macrophages [6], [36] *in vitro*, we elected to use 100 ng/ml to maximally-activate macrophage signaling pathways. After, monocytes were immunostained with an antibody specific for the human Tie2 receptor and analyzed by flow cytometry (**Figure 1A**). Our data suggests that CD14+ cells incubated in the absence of CSF1 for 24 hours express the Tie2 receptor similar to freshly-isolated CD14+ cells. In contrast, CD14+ monocytes cultured in the presence of CSF1 for 24 hours significantly increased Tie2 receptor expression (*p*<0.0001) (**Figure 1A**). Cell viability of all monocytes was confirmed by Trypan Blue staining (*data not shown*).

**Figure 1:** CSF1 up-regulates Tie2 receptor on CD14+ human monocytes. (**A**) CD14+ monocytes were isolated from whole blood using CD14+ microbeads. Cells were fixed and immunostained using anti-human Tie2 receptor antibody or isotype control antibody immediately following isolation (*Freshly isolated*) or after treated without (-*CSF1*) or with rhCSF1 (100 ng/ml) (+*CSF1*) for 24 hours. N = 10 per group and results represent the mean ± SEM of Tie2-positivity. (**B**) CD14+ monocytes treated with rhANG1 (100 ng/ml), rhANG2 (100 ng/ml) or a dose-response of rhCSF1 (0, 0.1, 1, 10, 100 ng/ml). ANG2 up-regulated Tie2 expression compared to ANG1 and CSF1 induces a dose-escalation of Tie2 on CD14+ monocytes. N = 10 per group and results represent the mean ± SEM of Tie2-positivity. (**C**) CD14+ monocytes were left untreated (*Utx*) or treated with rhANG2 (100 ng/ml) (*ANG2*), rhCSF1 (100 ng/ml) (*CSF1*), CSF1R neutralizing antibody alone, or pre-treated with the CSF1R Nab for 30 minutes prior to stimulation with rhCSF1 (100 ng/ml) (*CSF1R NAb+CSF1*) for 24 hours. ANG2- and CSF1-treatment significantly increased Tie2 expression while the CSF1R NAb abrogated this effect. N = 8 per group and results represent the mean ± SEM of Tie2-positivity by flow cytometry. (**D**) CD14+ monocytes were left untreated (*Untreated*), pre-treated with CSF1R NAb (40 µg or 80 µg) for 30 minutes then treated with rhCSF1 (100 ng/ml) (*CSF1R NAb+CSF1*), or with rhCSF1 (100 ng/ml) alone (*CSF1*) for 10 minutes. Western blot analysis indicates that the CSF1R NAb was effective at reducing Akt1 phosphorylation.

Next, we assayed the ability of low to moderate doses of CSF1 (0.1 to 10 ng/ml) to induce the differentiation of CD14+ monocytes to CD14+/Tie2+ TEMs. Importantly, dose escalation of CSF1 significantly increased Tie2 receptor expression on these cells (Trend Analysis for dose-dependency, *p* = 0.0003) (**Figure 1B**).

To compare the ability of CSF1 to induce Tie2 expression on CD14+ monocytes to known inducers of Tie2 expression on endothelial cells and TEMs, we cultured CD14+ monocytes in media containing angiopoietin-1 (ANG1) or angiopoietin-2 (ANG2). While ANG1 had no effect on Tie2 expression compared to untreated cells, ANG2 induced a significant increase in Tie2 expression (*p*<0.0001) but had fewer cells expressing the Tie2 receptor than with 100 ng/ml CSF1 alone (**Figure 1B** and *Figure S1*). This data suggests that tumor concentrations of CSF1 can induce a CD14+/Tie2- to CD14+/Tie2+ phenotype transition. To ensure that CSF1 was responsible for this Tie2+ transition, we pre-treated freshly-isolated CD14+ monocytes with a neutralizing antibody (NAb) to CSF1R for 30 minutes then treated with CSF1 and analyzed these cells for Tie2 expression. We found that pre-incubation with the CSF1R NAb significantly inhibited Tie2 expression on CD14+ cells compared to CSF1-treated cells after 24 hours, similar to Tie2 expression on untreated cells (*p*<0.0001) (**Figure 1C**). To illustrate the effect of the CSF1R NAb on CSF1 signaling pathway activation, CD14+ monocytes were pre-treated for 30 minutes with the CSF1R NAb followed by stimulation with CSF1 or left untreated for 10 minutes. Western blot analysis reveals a reduction in phosphorylated Akt in the presence of the antibody (**Figure 1D**).

### CSF1 enhances CD14+ monocyte migration towards ANG2

ANG2 binds the Tie2 receptor on endothelial cells allowing for the detachment of cellular adhesions and facilitating the migration of these cells during angiogenesis [37]. We next sought to determine if CSF1 up-regulation of the Tie2 receptor on CD14+ monocytes modulated migration towards ANG2. We pre-treated CD14+ human monocytes with or without 10 ng/ml CSF1 in the bottom well of Boyden chemotaxis chambers for 18 hours then washed the cells and replaced the media with FBS-containing media without or with a dose escalation of ANG2 in the top chamber. After 24 hours, the filters were inspected for migration of monocytes to the top chamber (chemotaxis) and cells blindly counted by microscopy. We observed that ANG2 stimulation alone induced significant migration at 100 ng/ml ANG2 compared to ANG2-free media (*p*<0.0001) (**Figure 2A**). Interestingly, pre-treating CD14+ monocytes with 10 ng/ml CSF1 significantly increased the number of migrating cells responsive to ANG2 compared to monocytes not pre-treated with CSF1 and reduced the significant migration response to ANG2 from 100 ng/ml without CSF1 to 1 ng/ml with CSF1 (*p* = NS without CSF1 pre-treatment and *p* = 0.0003 with CSF1 pre-treatment) (**Figure 2A**) suggesting that CSF1 pre-treatment increased the number of CD14+/Tie2+ cells during the 18 hour pre-incubation and resulted in a larger population cells able to respond to ANG2.

**Figure 2:** CSF1 pre-treatment augments the migratory response to ANG2 by CD14+ monocytes. (**A**) CD14+ monocytes were isolated and cultured in Boyden chemotaxis chambers in minimal media alone (*Media*), in media containing 0.1, 1, 10, 100 or 300 ng/ml rhANG2, or with the same ANG2 doses but first pre-treated for 24 hours with media containing 10 ng/ml rhCSF1 and analyzed for their migratory ability. A significant synergistic effect of CSF1 pre-treatment was first observed at 1 ng/ml rhANG2 and peaked at 100 ng/ml rhANG2. N = 8 and results represent the mean ± SEM of CD14+ monocyte migration through the Boyden chamber. (**B**) CD14+ monocytes were treated with rhANG2 (10 ng/ml) *(ANG2*) or rhCSF1 (10 ng/ml) (*CSF1*) alone, or pre-treated with rhCSF1 (10 ng/ml) for 24 hours, washed 3x, then treated with rhANG2 (10 ng/ml) for another 24 hours and transfected with a scrambled siRNA or an siRNA targeting the human Tie2 receptor. While ANG2 and CSF1 did not induce significant migration, the CSF1-pre-treated cells transfected with the scrambled siRNA migrated significantly more than those cells transfected with siRNA targeting Tie2. N = 8 and results represent the mean ± SEM of CD14+ monocyte migration through the Boyden chamber.

CD14+ monocytes express the receptor for CSF1 and migrate in response to CSF1 [38]. Because of this, we asked if TEM migration was a result of CSF1 or ANG2, the ligand for the Tie2 receptor. We again plated freshly-isolated CD14+ monocytes into the bottom wells of Boyden chambers and pre-treated with media containing CSF1 or media alone. Cells were washed after 18 hours of incubation and resuspended in fresh media. To analyze migration potential, CSF1 or ANG2 was added to the top chamber. We observed no difference in the ability of monocytes to migrate when cultured in CSF1- and ANG2-containing media (**Figure 2B**). This data suggests that the migratory response by CD14+ monocytes which differentiate to TEMs after pre-treatment with CSF1 is not attributed to CSF1 as a chemokine but is instead attributed to the presence of ANG2. To confirm that Tie2 receptor is regulating the migration of these cells, we transfected CD14+ monocytes with either a scrambled siRNA (*scrambled siRNA-GFP*) or a siRNA targeting the Tie2 receptor (*Tie2 siRNA-GFP*) for 18 hours. Subsequent to transfection, we separated CD14+ cells from dying cells and debris and into *positive* and *negative* fractions based on GFP expression using flow-assisted cell sorting followed by pre-treatment for 18 hours with CSF1. After, we replaced the media and added ANG2 in the top chamber for 4 hours. We found significantly more monocytes transfected with the scrambled siRNA in the top chamber compared to those cells transfected with the Tie2 siRNA (*p*<0.0001) suggesting that Tie2 receptor regulates the migration of these CD14+ monocytes (**Figure 2B**).

### CSF1 augments the angiogenic potential of CD14+ monocyte supernatants on HUVECs via Tie2 receptor up-regulation

Tumor angiogenesis requires endothelial cell proliferation, mobilization, and sprouting blood vessels. The human umbilical vein endothelial cell (HUVEC) tube branching assay is a method to analyze the angiogenic potential of endothelial cells *in vitro*. Conditioned supernatants from CSF1-treated human monocytes contribute to endothelial cell tube formation [13]. More specifically, conditioned supernatants from TEMs increase endothelial tube branching over that observed by conditioned supernatants from a TEM-depleted monocyte population [28]. Given our observation that CSF1 increases Tie2 receptor expression on CD14+ monocytes, we hypothesized that pre-treatment with CSF1 would induce macrophages to release factors which increase HUVEC tube branching and that blocking Tie2 receptor expression with an siRNA targeting monocyte Tie2 receptor would abrogate this effect. To determine the angiogenic potential of CSF1 up-regulation of the Tie2 receptor on monocytes, we isolated CD14+ monocytes from whole blood and differentiated to macrophages over five days using low-dose (5 ng/ml) rhCSF1. After starvation in minimal media, the cells were treated with either a neutralizing antibody for CSF1R or isotype antibody (40 µg/ml) for 1 hour prior to stimulation with CSF1 for 18 hours. The cells were then washed three times and treated with ANG2 for 24 more hours. The cell-free conditioned supernatants from these cells or minimal media alone, media containing ANG2 alone, media containing CSF1 alone, or media containing VEGF alone were used to culture 1.5×10^4^ human umbilical vein endothelial cells on growth factor-reduced Matrigel for 8 hours. The conditioned supernatants from the macrophages pre-treated with CSF1 induced significantly more HUVEC branch points than media containing CSF1, VEGF, and ANG2 alone (*p*<0.0001 for each condition). More importantly, pre-treatment of the macrophages with the CSF1R neutralizing antibody before CSF1 and ANG2 stimulation significantly reduced HUVEC branch points comparable to HUVECs cultured in media containing VEGF, media containing CSF1, and media containing ANG2 alone (*p*<0.0001) (**Figure 3A**).

**Figure 3:** Conditioned supernatants from CSF1-treated TEMs augments HUVEC branching. (**A**) Human monocytes were isolated from whole blood and differentiated to macrophages over five days using rhCSF1 (5 ng/ml). The cells were serum-starved in endotoxin-free RPMI containing polymyxin B (10 µg/ml) for 24 hours then treated with either a neutralizing antibody for CSF1R or isotype antibody (40 µg/ml) for 1 hour prior to stimulation with CSF1 (10 ng/ml) for 18 hours. The cells were then washed three times and treated with ANG2 (10 ng/ml) for 24 more hours. The conditioned supernatants from these cells (*CSF1/ANG2*; *CSF1R NAb/CSF1/ANG2*) or minimal media alone, (*minimal*), media containing ANG2 alone (10 ng/ml) (*ANG2*), media containing CSF1 alone (10 ng/ml) (*CSF1*), or media containing VEGF (10 ng/ml)(*VEGF*) were used to culture 1.5×10^4^ human umbilical vein endothelial cells (HUVEC) on growth factor-reduced Matrigel for 8 hours. Digital images were captured to determine HUVEC branching. The number of branches was quantified in a blinded manner per field. CSF1, VEGF, and ANG2 each stimulated significantly more branch points from the HUVECs than minimal media. The conditioned media from the macrophages pre-treated with CSF1 induced significantly more branch points than CSF1, VEGF, and ANG2 treatment alone and pre-treatment of the macrophages with the CSF1R neutralizing antibody significantly reduced branch points comparable to media containing VEGF, CSF1, and ANG2 alone levels. N = 5 and results represent the mean ± SEM of HUVEC branch points. (**B**) In the same manner as above, human monocytes were differentiated to macrophages over five days and serum-starved for 24 hours. The cells were transfected with a siRNA targeting human Tie2 receptor (50 nM) or a scrambled siRNA (50 nM) for 24 hours. The macrophages were washed three times with PBS and then treated with CSF1 (10 ng/ml) for 18 more hours. These conditioned supernatants were collected and used to culture HUVEC cells grown on growth factor-reduced Matrigel for eight hours to detect branch points. Digital images were captured to determine HUVEC branching. The macrophages pre-treated with CSF1 then ANG2 (*CSF1/ANG2*) induced a significant number of branch points compared to HUVEC cultured in media alone (*Media*). The conditioned supernatants from the macrophages transfected with siTie2 then treated with CSF1 then ANG2 (*Tie2 siRNA/CSF1/ANG2*) had significantly less branch points than the CSF1-conditioned supernatants and similar to the minimal conditions. The macrophages transfected with the scrambled siRNA and pre-treated with CSF1 then ANG2 (*scrmbsiRNA/CSF1/ANG2*) induced significantly more branch points than the conditioned supernatants from the siTie2 samples but still significantly less than the CSF1-conditioned media. N = 5 and results represent the mean ± SEM of HUVEC branch points. (**C**) CD14+ monocytes were left untreated (*UTX*) or treated with CSF1 (100 ng/ml) (*CSF1*), ANG2 (100 ng/ml) (*ANG2*), or the combination CSF1 (100 ng/ml) and ANG2 (100 ng/ml) (*CSF1+ANG2*) for 48 hrs. RT-PCR analysis for mRNA expression of the following angiogenic factors was performed: VEGF, uPA, COX2, TNFα, MMP2, MMP7, and MMP9. Data is represented as relative expression for each target mRNA relative to GAPDH housekeeping mRNA. VEGF, uPA, and COX2 mRNA were all significantly increased in CD14+ monocytes treated with CSF1+ANG2 compared to untreated CD14+ monocytes. Each condition was repeated at least 3 times (N = at least 3 and results represent the mean ± SEM for relative mRNA expression).

Next, to demonstrate a casual role for the Tie2 receptor expressed on these monocytes regarding increased angiogenic potential on endothelial cells, we isolated and transfected CD14+ human monocytes with a scrambled siRNA or siRNA targeting human Tie2 receptor as described above followed by treatment with CSF1 then ANG2 as before. The cell-free supernatants were collected and used to culture HUVEC on growth factor-reduced Matrigel for 8 hours followed by tube branching analysis. The role of the Tie2 receptor on HUVEC branching was confirmed as conditioned supernatants from CD14+ monocytes transfected with the Tie2 siRNA induced significantly less HUVEC branching compared to conditioned media from CSF1 then ANG2 treated cells (*p*<0.0001) and conditioned supernatants from monocytes transfected with the scrambled control siRNA (*p*<0.0001) (**Figure 3B**). This data confirms the importance of the Tie2 receptor on the angiogenic function of CD14+/Tie2+ cells. The factors produced by CSF1-induced Tie2 receptor upregulation driving this effect is being investigated in our laboratory.

TEMs are reported to augment tumor angiogenesis by producing pro-angiogenic factors similar to M2-type cells as well as provide structural support by migrating proximal to vessels [63]. Because we found that supernatants from CSF1/ANG2-stimulated CD14+ monocytes augmented vessel branching from HUVECs, we investigated gene expression differences of a signature set of genes which contribute to angiogenesis. We treated CD14+ monocytes with CSF1, ANG2, or the combination CSF1/ANG2, or left them untreated in media containing 1% FBS for 48 hours then analyzed by RT-PCR for differential expression of VEGFA, uPA, COX2, TNFα, MMP2, MMP7, and MMP9. We found significant differences from CSF1/ANG2 combination treated cells in VEGF, uPA, and COX2 mRNAs, but not in TNFα, or MMPs-2, -7, and -9 mRNAs (**Figure 3C**).

### CSF1 treatment increases the tumor F4/80+/Tie2+ TEM population and augments angiogenesis while having no effect on tumor growth

High serum levels of CSF1 correlate with poor prognosis and increased metastasis in patients with breast cancer[15], [39] Further, increased levels of CSF1 in the tumor microenvironment correlate with increased vessel density and metastasis[20], [21]. Because TEMs are reported as being one of the most potent cell types in supporting vascularization, and because we found that CSF1 up-regulates Tie2 receptor expression on CD14+ human monocytes, we asked if CSF1 treatment would expand the number of tumor TEMs and alter angiogenesis in a mouse model of breast cancer. PyMT tumor cells were injected subcutaneously into the number 4 mammary fat pad of wild type C57/Bl6 mice and the tumors were grown until palpable. After, intratumoral injections with PBS, CSF1, a CSF1R neutralizing antibody (NAb), CSF1R NAb pre-treatment in combination with CSF1, isotype IgG antibody, or isotype IgG antibody pre-treatment in combination with CSF1 were performed every other day for two weeks. Tumor growth data suggests no significant increase in tumor growth rate from tumors treated with CSF1 compared to PBS (*data not shown*).

Upon sacrifice, fresh tumors were collected, homogenized using collagenase, immunostained with F4/80 and Tie2 receptor antibodies and subjected to flow cytometry for the percent of total F4/80+ cells and percent of F4/80+/Tie2+ TEMs relative to tumor cells. CSF1 treatment induced a significantly higher percentage of F4/80+/Tie2+ TEMs (*p* = 0.0003) than the percentage of overall tumor F4/80+ cells (**Figure 4A**) while a neutralizing antibody to CSF1R abrogated this effect. These data suggest that CSF1 contributes more to the expansion of the population of tumor TEMs than overall F4/80+ cells. To corroborate the flow cytometry data, we immunostained +/- CSF1 treated tumors with CD31, F4/80, or Tie2 antibodies and analyzed by confocal microscopy and found differences in both overall F4/80+ infiltration as well as an increase in F4/80+/Tie2+ cells (TEMs) in the CSF1-treated tumors (**Figure 4B** **).**

**Figure 4:** CSF1 has no effect on tumor growth but increases percent tumor TEMs and augments angiogenesis. (**A**) After two weeks of treatment, tumors were removed, homogenized and immunostained with antibodies specific for F4/80 and Tie2 to identify total F4/80+ cells and F4/80+/Tie2+ cells (Tie2-expressing macrophages, TEMs). While there was a marked increase in total F4/80+ macrophages with CSF1 treatment, the percent of F4/80+/Tie2+ TEMs was significantly increased in response to CSF1 suggesting a regulatory role for CSF1 in expanding the TEM population. N = 5 mice per group and results represent the mean ± SEM of total F4/80+ and F4/80+/Tie2+ TEMs within the tumors. (**B**, *top and bottom left*) PyMT tumors without CSF1 treatment and (*top and bottom right*) with CSF1 treatment immunostained with CD31 for blood vessels, F4/80 for macrophages, Tie2 for F4/80+/Tie2+ TEMS, and DAPI. Confocal images (using 60× objective (*top*) and with 3× zoom (*bottom*) suggest an increase in both F4/80 macrophages and F4/80+/Tie2+ TEMS in the CSF1-treated tumors. *Multiply overlap* indicates those areas where F4/80 and Tie2 positivity overlap. Individual stains are in *Supplementary* *Figure 3*. (**C**, *top*) Orthotopically implanted PyMT mammary tumors in wild type C57Bl/6 female mice were allowed to become palpable then intraperitoneally treated with PBS (*PBS*), CSF1 (100 ng in 100 µls) (*CSF1*), a neutralizing antibody for the CSF1R (50 mg/kg) 4 hours prior to CSF1 treatment (100 ng in 100 µls) (*CSF1R NAb+CSF1*), the CSF1R antibody alone (*CSF1R NAb*), an isotype antibody (50 mg/kg) 4 hours prior to CSF1 (100 ng in 100 µls) treatment (*CSF1+IgG*), or the isotype antibody alone (*IgG*) three times per week for two additional weeks. The tumors were immunostained with a CD31-Alexa Flour 546 antibody to recognize endothelial cells that comprise blood vessels. Qualitatively, CSF1 treatment increased the percent of CD31-postitive pixels per high powered field compared to PBS treated tumors, while the neutralizing antibody to CSF1R suppressed the CSF1 effect on angiogenesis. (**B**, *bottom*) Quantitatively, the percent of CD31+ pixels per high powered field were quantified as blood vessels (angiogenesis) using Adobe Photoshop histogram analysis. CSF1 treatment significantly increased CD31-positive pixels (angiogenesis) compared to PBS. The neutralizing antibody for CSF1R significantly reduced the ability of CSF1 to up-regulate angiogenesis. N = 5 mice per group and results represent the mean ± SEM of percent CD31-positive pixels per high powered field (HPF).

Because macrophages drive tumor progression and angiogenesis, we analyzed sections of these tumors for increased blood vessel formation in response to CSF1. We observed significantly more CD31+ blood vessels in the tumors treated with CSF1 compared to those tumors treated with PBS (*p*<0.0001) or pre-treated with the neutralizing antibody toward CSF1R plus CSF1 treatment (*p*<0.0001) (**Figure 4C**). These data highlight the role of CSF1 in tumor angiogenesis.

### High serum levels of CSF1 expands the circulating TEM population

Because we observed increased numbers of TEMs within the tumors of the CSF1-treated mice, we hypothesized that CSF1 may be inducing recruitment of TEM progenitors from bone marrow. Because breast cancer patients can have higher than normal levels of serum CSF1[39], [40], we emulated these serum levels of CSF1 in non-tumor bearing wild type mice to see if in the absence of a tumor that CSF1 could expand circulating levels of TEMs. We intravenously injected PBS or CSF1 at a concentration which emulates human breast cancer patients. Flow cytometry analysis revealed no difference between treatment groups in CD45+/Tie2+ cells from the bone marrow, described as TEM bone marrow precursors[24], [27] (**Figure 5**). Interestingly, we observed a significant reduction in circulating CD11b+/CD31-/Gr-1^lo^/Tie2- monocytes (*p*<0.0001) and a significant increase in circulating CD11b+/CD31-/Gr-1lo/Tie2+ cells (TEMs) (*p*<0.0001) with CSF1 treatment (**Figure 5**). This data suggests that serum CSF1 can regulate TEM expansion in circulation and not solely once monocytes enter the tumor proper.

**Figure 5:** CSF1 expands the TEM population in peripheral blood. To reach serum levels of CSF1 similar to breast cancer patients and determine that effect on TEM expansion, PBS or CSF1 (20 ng/ml) was intravenously injected into non-tumor bearing wild type C57Bl/6 female mice every other day for a total of three treatments. Bone marrow and atrial blood was collected and immunostained with CD45 and Tie2 antibodies (for bone marrow) or CD11b, CD31, Gr-1, and Tie2 antibodies (for blood). There was no difference in the percentage of TEMs in the bone marrow of the PBS- and CSF1-treated mice. In peripheral blood, CSF1 treatment significantly reduced the percent of CD11b+/CD31+/Gr-1lo/Tie2- cells while significantly increasing CD11b+/CD31+/Gr-1lo/Tie2+ TEMs. N = 5 mice per group and results represent the mean ± SEM of percent total CD45+ and CD45+/Tie2+ cells from bone marrow, and the percent of CD11b+/CD31-/Gr-1lo/Tie2- and CD11b+/CD31-/Gr-1lo/Tie2+ TEMs in peripheral blood.

### CSF1 and HIF pathways can individually and synergistically regulate Tie2 receptor expression on TEMs in an oxygen-independent manner

The hypoxia inducible factor, HIF-1α, has been linked to CSF1 and PI3 kinase/AKT signaling pathways [41]–. Further, macrophages reside in hypoxic patches in solid tumors. We asked if HIF-1α was involved in the CSF1-induced increase in Tie2 receptor expression on TEMs. We differentiated bone marrow-derived macrophages from HIF-1α*^fl/fl^*/LysMcre and LysMcre (wild type) mice and stimulated these cells with PBS or CSF1. After 24 hours, we analyzed the macrophages for expression of Tie2 receptor by flow cytometry. We found no difference in the percent of F4/80+ macrophages expressing Tie2 receptor in the PBS-treated wild type LysMcre cells compared to HIF-1α-deficient cells (**Figure 6A**). In the CSF1-treated cells, we found that the loss of HIF-1α significantly inhibited the ability of these F4/80+ macrophages to express Tie2 receptor (*p*<0.0001) (**Figure 6A**). These data suggest an oxygen-independent role for HIF-1α in CSF1 augmentation of TEMs.

**Figure 6:** CSF1 and HIF pathways independently and synergistically regulate Tie2 receptor expression on monocytes. (**A**) Bone marrow-derived macrophages were differentiated from age-matched wild type LysMcre and HIF-1α*^fl/fl^*/LysMcre mice over five days in non-adherent tubes. After, the cells were serum-starved in endotoxin-free RMPI for 24 hours. The cells were treated with PBS or CSF1 (100 ng/ml) for 24 hours followed by immunostaining with antibodies specific for F4/80 and Tie2 receptor. CSF1 induced an increase in F4/80+/Tie2+ cells over PBS-treated cells from the macrophages derived from the bone marrow of wild type LysMcre mice. The macrophages derived from the HIF-1α*^fl/fl^*/LysMcre bone marrow and treated with CSF1 had a significantly smaller percentage of F4/80+ Tie2+ cells than those from the wild type mice. N = 5 per group and results represent the mean ± SEM of percent F4/80+/Tie2+ cells of total F4/80+ cells. (**B**) Macrophages were derived from the bone marrow of wild type female mice over five days in non-adherent tubes. The cells were serum-starved in endotoxin-free RMPI for 24 hours. The cells were pre-treated with DMSO (*vehicle*), the PI3 kinase/Akt inhibitor LY294002 (50 µM) (*LY294002*), the MEK inhibitor U0126 (10 µM) (*U0126*), or the NF-Kb inhibitor PDTC (100 µM) (*PDTC*) for 30 minutes. After, the cells were treated with CSF1 (100 ng/ml) (*Vehicle+CSF1*), LY294002+CSF1 (100 ng/ml) (*LY294002+CSF1*), U0126+CSF1 (100 ng/ml) (*U0126+CSF1*), or PDTC+CSF1 (100 ng/ml) (*PDTC+CSF1*) or left untreated for 24 hours followed by immunstaining with antibodies specific for F4/80 and Tie2. CSF1 induced an increase in the percent of F4/80+/Tie2+ cells compared to vehicle alone. The inhibitors LY294002, U0126, and PDTC alone had no effect on TEM levels. LY294002 pre-treatment significantly reduced the percent of TEMs regulated by CSF1 while U0126 and PDTC had no effect on CSF1 expansion of TEMs. Results represent the mean ± SEM of percent F4/80+/Tie2+ cells of total F4/80+ cells. (**C**) Bone marrow-derived macrophages were differentiated from age-matched wild type LysMcre and HIF-1α*^fl/fl^*/LysMcre mice over five days in non-adherent tubes. After, the cells were serum-starved in endotoxin-free RMPI for 24 hours. The cells were then pre-treated with DMSO or LY294002 (50 µM) for 30 minutes followed by CSF1 (100 ng/ml) (*LY294002+CSF1*) or not (*vehicle*) for 24 hours and then immunostained with antibodies specific for F4/80 and Tie2. The macrophages derived from HIF-1α*^fl/fl^*/LysMcre mice in combination with the PI3 kinase inhibitor LY294002 significantly reduced the percent TEMs to that similar to untreated levels. N = 5 per group and results represent the mean ± SEM of percent F4/80+/Tie2+ cells of total F4/80+ cells.

Because a considerable percentage of F4/80+ macrophages still demonstrated Tie2-positivity in the HIF-1α KO macrophages treated with CSF1 compared to vehicle treatment, we asked which signaling pathway downstream of the CSF1R regulated Tie2 receptor expression on TEMs. We pre-treated with the appropriate vehicle or the PI3 kinase inhibitor LY294002 (50 µM), the MEK inhibitor U0126 (10 µM), or the NF-κB inhibitor PDTC (100 µM) for 30 minutes then stimulated with CSF1 or not for 24 hours. CSF1 has been reported to activate all three of these signaling pathways [5], [6], [36], [44], [45]. Of the three inhibitors assayed, only the inhibitor abrogating PI3 kinase activity (LY294002) significantly suppressed the percentage of TEMs generated by CSF1 stimulation (*p*<0.0001) (**Figure 6B**). Further, when we assayed wild type or HIF-1α KO macrophages in the absence or presence of LY294002, we found that the ability of CSF1 to augment Tie2 receptor expression was abolished to vehicle-treated levels (*p* = 0.05) (**Figure 6C**). Taken together, these data suggest that CSF1 and HIF-1α pathways regulate Tie2 receptor expression on TEMs independently, and that there is some level of synergy between to the pathways regulating this activity. Further analysis of this regulation is ongoing in our laboratory.

## Discussion

This paper establishes a novel role for CSF1 in regulating Tie2 receptor expression on macrophages *in vitro* and *in vivo* in a model of murine breast cancer. The impetus for this study stemmed from independent reports that CSF1 and TEMs increase tumor vascular density and pulmonary metastasis in tumors [20], [21], [23], [24], [26]. We hypothesized that because CSF1 can differentiate macrophages with a pro-tumor M2 phenotype, that CSF1 might also be differentiating a subpopulation of Tie2-expressing monocytes/macrophages (TEMs) that can be recruited by angiopoietins into breast tumors.

Although not classified as M2 macrophages, TEMs maintain a pro-angiogenic profile [27], [28]. For example, co-injection of isolated TEMs with glioma tumor cells increased vascular area over those glioma cells injected with Tie2 receptor negative monocytes [23]. On endothelial cells, the expression of the Tie2 receptor is dynamic, increasing during hypoxia through binding of its ligand, ANG2, resulting in stimulation of transcription factors Gata3 and Ets-1 [46], [47]. Our current study demonstrates that CSF1 treatment induces increased pro-angiogenic activity on both human and mouse monocytes when the Tie2 receptor is expressed and that the Tie2 receptor is responsible for this activity. We examined the functional consequences of an expanded TEM population as it pertains to monocyte migration as CSF1 augmented Tie2 receptor-driven migration of monocytes toward ANG2. Previous studies show that the Tie2 receptor is required for TEM migration towards ANG2 and we found that pre-treatment with CSF1 decreases the threshold of ANG2 required for this response and increases the number of migrating cells, *in vitro*. This study is of importance because ANG2 levels are expressed in a variety of solid tumors, including breast cancer [48]–[52]. In fact, although ANG2 overexpression increases the number of TEMs in breast cancer [28], monoclonal antibodies blocking ANG2 inhibits TEM interaction with blood vessel endothelial cells in a PyMT mouse model of breast cancer, limiting their supportive nature and pro-angiogenic function on endothelium [26]. We found that pre-treatment of human CD14+ monocytes with CSF1 resulted in Tie2 receptor overexpression and a significant increase in endothelial cell branch points when cultured with conditioned supernatants from these TEMs. In both of our TEM functional studies, antibody neutralization of the CSF1R and knockdown of the Tie2 receptor on monocytes using siRNA targeting Tie2 abrogated the synergistic effect of CSF1 pre-treatment and ANG2.

Because we found expanded TEM populations and enhanced soluble factor release that activated endothelial cell function with CSF1 pre-treatment, we next asked what effects exogenous CSF1 treatment would have in a PyMT tumor model of breast cancer. We showed that while intratumoral administration of CSF1 did not significantly increase the overall percent of F4/80+ macrophages in these tumors, the percentage of F4/80+/Tie2+ TEMs was significantly augmented. As stated previously, TEMs are cells of a pro-angiogenic phenotype which express high levels of VEGF, MMPs, cathepsin B, and thymidine phosphorylase which break down extracellular matrix facilitating angiogenesis [28]. Likewise, CSF1 increases expression of these same factors from macrophages *in vitro* as well as in models of breast cancer [13], [53]–[56]. We observed changes in vascular density assayed by CD31-positivity in the tumors treated with CSF1 corresponding to augmentation of the TEM population.

Tumor cells express high levels of CSF1 as shown in the serum of patients with various cancer types [5], [13], [32], [57]. Serum CSF1 mobilizes bone marrow monocyte precursor cells to release and migrate to the tumor site, as well as activates and differentiates these cells into macrophages while skewing their phenotype in support of a Th2 response [58]. In turn, these macrophages produce epidermal growth factor (EGF) which enhances tumor cell proliferation [59]. This EGF/CSF1 paracrine loop increases tumor cell intravasation and, in fact, it has been shown that tumor cells and macrophages alternate leaving the tumor into circulation [59], [60]. Given the functional similarities between CSF1 effects on monocytes and TEM function and our data showing a connection between CSF1 and TEM expansion, further work to explore a link between TEMs and mechanisms regulating tumor angiogenesis and progression is warranted. Further, ANG2-stimulated monocytes produce immunoregulatory IL-10, suppressing T cell proliferation *in vitro* [29]. In tumors, T cells produce IL-4 which primes macrophages to produce EGF to augment tumor cell proliferation [61].

The fact that we observed an expansion of the CD11b+/CD31-/Gr-1^lo^/Tie2+ population without an overall expansion of total CD11b+/CD31-/Gr-1^lo^ monocytes in circulation when administering CSF1 to levels similar to that of breast cancer patients[15] suggests that CSF1 can actuate TEM differentiation from monocytes already in circulation which have potential to migrate to the tumor and become M1, tumor-fighting cells, yet are usurped by high serum levels of CSF1 to induce Tie2 receptor expression and adopt an M2-like, tumor supporting phenotype.

In summary, we hypothesized that CSF1, which induces an M2 macrophage phenotype, could expand a subpopulation of macrophages that also express the Tie2 receptor, canonically known to be expressed on endothelial cells. This data supports a recent finding from He et al 2012 that describes endothelial cell-derived CSF1 differentiation of naïve hematopoietic cell precursors into Tie2/CD206-expressing macrophages in co-culture [62]. We found that CSF1 differentiated TEMs and that these cells are more responsive to ANG2 stimulation resulting in increased cell migration and pro-angiogenic potential on HUVECs. Further, we found that CSF1 treatment in a mouse model of breast cancer increases tumor angiogenesis but had limited effect on tumor growth. This activity was determined to be regulated by synergistic contribution of each the PI3 kinase pathway and HIF pathway in an oxygen-independent manner. The importance of this study is highlighted by our data suggesting that high serum levels of CSF1 in breast cancer patients may be responsible for increasing the number of circulating monocytes recruited to tumors and support their progression.

## Supporting Information

Figure S1 Flow cytometry of TIE2 receptor expression on monocytes.
(TIF)

Figure S2 siRNA for TIE2 receptor mRNA knock down.
(TIF)

Table S1 RT-PCR primers.
(TIF)
